# Effects of school-based physical activity on volition in exercise, sleep quality and internet addiction in Italian adolescents

**DOI:** 10.1016/j.heliyon.2024.e32129

**Published:** 2024-05-29

**Authors:** Francesca Greco, Federico Quinzi, Maria Cristina Papaianni, Loretta Francesca Cosco, Cristina Segura-Garcia, Gian Pietro Emerenziani

**Affiliations:** a Department of Movement, Human and Health Sciences, University of Rome “Foro Italico”, Rome, RM, Italy; b Department of Experimental and Clinical Medicine, University “Magna Græcia” of Catanzaro, CZ, Italy; c Italian Ministry of Education, Crotone, KR, Italy; d Department of Movement Sciences and Wellness, University Parthenope, Naples, NA, Italy; e Department of Health Sciences, University Magna Graecia of Catanzaro, CZ, Italy

**Keywords:** Non-communicable diseases, Exercise, Body composition, Healthy lifestyles, Sedentary behavior

## Abstract

School-settings represent ideal context to promote healthy habits as in adolescence most risk factors may occur or intensify leading to the adoption of unhealthy lifestyles. Thus, a deeper understanding of the factors promoting healthy lifestyles in adolescents is of utmost importance.

This observational study aims to investigate: 1) gender-related differences in physical activity (Physical Activity Questionnaire for Adolescets – PAQ-A), sleep quality (Pittsburgh Sleep Quality Index - PSQI) and internet addiction (Internet Addiction Test – IAT) levels and Volition in Exercise (VE); 2) the relationship between PAQ-A and VE, PSQI and IAT; 3) the effects of a five-month (T0; T5) school-based physical activity (PA) intervention on the above-mentioned factors. PAQ-A,VE, PSQI and IAT were assessed before (T0) and after (T5) a school-based PA intervention. The PA intervention consisted of coordinative exercises and team sports performed for 1 h twice a week. At T0, girls showed lower PAQ-A, PSQI scores, lower volition facilitators (“self-confidence” and “coping with failure”) and higher volition inhibitor (“postponing training”) than boys. Significant correlations were observed for volition factors an IAT in males and volition and PSQI and IAT in females. After the PA intervention (T5), “postponing training” and “self-confidence” factors were reduced compared to T0.

Exercise specialists should consider gender differences in volition in exercise factors during a school-based PA to plan and realize PA protocols aiming at maximizing exercise adherence to tackle sedentary behaviors in adolescents.

## 1 Introduction

Non-communicable diseases (NCDs; e.g., type 2 diabetes, cancers and cardiovascular diseases) are the leading cause of mortality and poor quality of life worldwide [1] Each year, 17 million people die from a NCD before age 70 and, cardiovascular diseases account annually for most deaths, followed by cancers, chronic respiratory diseases, and diabetes [2]. The global financial burden of NCDs is staggering. Indeed, it has been estimated that in 2030 the global costs of NCD will reach 13 trillion dollars [3]. The WHO recognized four major lifestyle-related risk factors for the onset of NCDs: physical inactivity, tobacco use, unhealthy diets and the harmful use of alcohol [4]. Notably, these risk factors are not mutually exclusive, and their co-occurrence may exponentially raise the risk of NCDs. Noteworthy, among the different stages of life, it is in adolescence that these risk factors may occur or intensify leading to the adoption of unhealthy lifestyles [5]. Available evidence suggests that physical inactivity and low fruit/vegetables consumption are the two most prominent lifestyle-related risk factors for NCDs in adolescents in both sexes [5]. Adolescents are primarily affected by internet addiction which is considered a behavior-based addiction that could influence both physical and mental health [6,7]. Specifically, internet addiction refers to an excessive or poorly controlled behavior to access the internet leading adolescents to use it day and night without worrying about its side effects [6]. A strong relationship exists between physical activity (PA), internet addiction and sleep quality [8,9]. Indeed, adolescents with low PA and high screen-based sedentary behavior scores tend to prefer internet use than those with high levels of PA and low screen-based sedentary behavior scores [8]. Therefore, maintaining sufficient PA levels and reducing screen-based sedentary behavior may contribute to reduce their internet addiction. Positive effects of PA on sleep quality were observed when PA is performed at moderate-intensity rather than high-intensity PA [9] with male adolescents reporting better sleep quality than females [10].

Among the modifiable unhealthy behaviors, physical inactivity has been deemed accountable for approximately 6–10 % of the major NCDs [11]. Scientific evidence highlighted the benefits of PA in children and adolescent's health [12,13]. The WHO recommends an average of 60 min per day of moderate-to vigorous-intensity, across the week with the implementation of strength exercise at least 3 days a week [13]. However, a recent review showed insufficient PA levels in children and adolescents, lower levels of PA among girls, and attenuation of PA levels across the lifespan [14]. Therefore, the promotion of PA is a key factor to counteract negative lifestyle behaviors among adolescents. In this scenario, the school environment seems to be an ideal setting for the promotion of PA, since a large number of adolescents may be reached simultaneously. Previous studies settled in a school-based environment have shown that educational interventions on lifestyle, nutrient adequacy, and diet quality as well as the implementation of PA, may facilitate the promotion of healthy habits in children and adolescents [15,16]. Therefore, school setting may provide opportunities to be physically active, since adolescents may participate in PA classes and may be encouraged to establish a long-lasting healthy lifestyle.

It is well established that both psychological and motivational factors may influence the participation of individuals in regular PA [17,18] with girls showing more barriers than boys [19]. However, together with motivational processes that lead to the intention of a behavioral change, volitional processes are deemed essential to transform intention into concrete action, leading to the actual behavior [18]. The concept of volition goes beyond self-confidence [20] and locus of control [21] and refers to an individual's self-regulatory mental processes that are responsible for taking and maintaining a desirable action (e.g., exercising regularly), even when this action is exposed to internal and external resistance [18]. Indeed, volition in exercise is a psychological construct that deeply explains why individuals either maintain or refrain from exercising regularly. To date, no data is available regarding the effects of school-based PA on volition in exercise, internet addiction and sleep quality in adolescent students. Taking into account the above-mentioned considerations, the implementation of policies aiming at increasing the amount of PA among adolescents is a strategic asset to pursue health promotion and to counteract the late onset of NCDs.

Therefore, this study aims to delve into the relationship among volition in exercise, sleep quality, and internet addiction and, to evaluate the effects of a school-based PA intervention on the above-mentioned variables. The results of this study may be helpful to plan and realize specific interventions promoting lifestyle changes in adolescents to prevent the onset of NCDs.

## 2 Materials and methods

### 2.1 Participants

For this study, 153 healthy adolescents (101 girls, 52 boys, mean age: 15.61 ± 1.33 years – Age range 14–19 years old) were recruited. All participants attended a local high school in southern Italy. Gpower software 3.1 [22] was used to calculate a priori the sample size (statistical power (β = 0.80) statistical significance (α = 0.05); medium effect size of 0.25). Participants were included in the study if they had no contraindication to the practice of PA and had no upper or lower limb injuries in the twelve months preceding the study. They were excluded from the study if they had cardiac pacemakers or prosthetic implants preventing the evaluation of their body composition.

After being informed of the aims, risks and benefits of the study, participants gave their assent and their legal guardians, in case of minors, gave their consent to participate in this study by signing the written informed consent approved by the Italian Ministry of Education (MUR; protocol number: 0005570). All the procedures detailed in the following paragraphs comply with the Declaration of Helsinki on studies on human participants.

### 2.2 Experimental procedures

Participants were evaluated at baseline (T_0_) and five months later after a school-based PA intervention (T_5_). All study procedures were carried out in a high school setting.

#### 2.2.1 Anthropometric and body composition characteristics

Anthropometry and body composition were assessed in all participants. Specifically, participants’ height was measured using a stadiometer to the nearest 0.01 m while body composition was evaluated using a hand-to-foot bioelectrical impedance instrument while participants stood in an upright position (InBodyR20, Seoul, Korea). This device enables an accurate evaluation of Muscle Mass (MM), Fat Mass (FM), Body Mass Index (BMI), percentage of Fat Mass (% FM) and Basal Metabolic Rate (BMR).

#### 2.2.2 Questionnaires

Volition was assessed using the Volition in Exercise Questionnaire (VEQ – [18]. The Italian version of this questionnaire includes eighteen items scored on a rating ranging from zero “it doesn't match at all” to three “exactly matches” [23]. The VEQ is composed of four volitional inhibition factors (VI), which hamper an individual's goal achievement, and two volitional facilitation factors (VF), which facilitate goal attainment. The VI of the VEQ are Reasons, Postponing Training, Unrelated Thoughts, and Approval from Others, whereas the VF are Self-Confidence, and Coping with Failure.

Behavioral factors were assessed through the administration of different questionnaires. Specifically, PA levels were assessed using the Physical Activity Questionnaire for Adolescents (PAQ-A). This questionnaire has been developed to assess general levels of PA in high school students 14–19 years of age. The PAQ-A can be administered in a classroom setting and provides a summary of PA score derived from eight items, each scored on a five-point Likert scale. This questionnaire assesses the PA performed in the last week preceding its administration [24], and has been used in other studies for the adolescent population of southern Italy [25].

Sleep quality was assessed using the Pittsburgh Sleep Quality Index (PSQI - [26]. This questionnaire assesses several sleep issues that may affect sleep quality. It consists of nineteen items investigating quantitative characteristics of sleep [26]. A version of this questionnaire has been validated for the Italian population [27].

The Italian version of the Young's Internet Addiction Test (IAT) was administered to the participants to quantify their Internet addiction risk. The IAT comprises twenty items, each scored on a one to five scale [28]. The Italian version of this questionnaire has been shown to have good psychometric properties [29].

#### 2.2.3 School-based intervention

The school-based PA intervention was administered during the PE classes and consisted of coordination exercises, encompassing eye-hand and eye-foot coordination exercises and team sports, encompassing volleyball, football, futsal, and basketball. The school-based PA intervention was carried out bi-weekly for 1 h and lasted for 5-months. The teacher monitored PA intensity using the rate of perceived exertion scale [30] in each class session throughout the five months of intervention. Exercise intensity was maintained moderate for coordinative exercises and vigorous for team sports activities.

### 2.3 Statistical analysis

Statistical analysis was carried out using IBM®SPSS version 23.0 statistical software (SPSS Inc., Chicago, IL, USA). The normal distribution of the dependent variables was verified using the Shapiro-Wilk test. This test showed that most of the variables had a skewed distribution, and therefore a non-parametric statistical approach has been adopted. In the following paragraphs, variables will be presented as median and interquartile range (IQR). For all statistical analyses, the significance level was set at p = 0.05. Gender differences at baseline (T_0_) in body composition parameters, and in behavioral factors were evaluated using the Mann-Whitney *U* Test for independent samples. To investigate the association between the abovementioned variables Spearman's Rho was carried out separately for girls and boys. Body composition parameters and behavioral factors were compared using the Wilcoxon Signed Rank Test before (T_0_) and after intervention (T_5_) intervention. Due to COVID-19 restrictions, a subgroup of adolescents (*n* = 43) completed the entire assessment at T_5_.

## 3 Results

The statistical analysis revealed that boys had significantly higher MM and BMR than girls (all *p-values* < 0.001), whereas girls had higher %FM (*p* < 0.001) than boys. There was no significant difference in BMI between genders (*p* = 0.55). The Mann-Whitney *U* test carried out on the PAQ-A showed that boys were more active than girls (p < 0.01). Among the volition inhibitors, the only factor differing between the two genders was “postponing training” (*p* < 0.01) with boys showing lower values than girls, whereas the other volition inhibitors did not differ between the genders (all *p-values* > 0.05). Concerning the volition facilitators “self-confidence” and “coping with failure”, a significant effect of gender was observed with higher scores in boys compared to girls (*p* < 0.001 and *p* = 0.027, respectively). In girls, sleep quality, as assessed via the PSQI, was lower than in boys (*p* = 0.019). No significant difference between girls and boys was observed for the internet addiction test (IAT; *p* = 0.174). Table 1 shows body composition and behavioral factors for girls and boys at T_0_.

**Table 1:** Body composition and behavioral factors across gender.

	Girls (*n* = *101*)	Boys (*n* = *52*)	Total (*n* = *153*)
Age [years]	15.0(2.0)	16.0(2.0)	16.0(1.0)
Height [m]	1.58(0.08)	1.71(0.11)*	1.62(0.14)
Mass [kg]	55.7(14.8)	70.9(18.9)*	60.6(20.0)
Muscle Mass [kg]	20.6(4.2)	30.7(18.9)*	22.7(9.6)
Fat Mass [kg]	18.4(9.7)^§^	13.6(11.0)	16.6(10.1)
BMI [kg/m^2^]	20.34(3.67)	21.47(4.30)	20.76(4.34)
Fat Mass [%]	32.8(9.8)^§^	18.4(13.2)	28.3(14.9)
BMR [kcal]	1206.0(139.0)	1579.5(300.3)*	1274.0(322.0)
PAQ-A	1.76(0.64)	2.45(1.04)*	1.92(0.88)
VEQ - inhibitors			
*Reasons*	1.00(2.00)	2.00(2.00)	1.00(1.00)
*Postponing training*	1.25(2.00)§	0.75(1.00)	0.75(2.00)
*Unrelated thoughts*	0.67(2.00)	0.67(1.00)	0.67(2.00)
*Approval from others*	1.00(1.00)	1.33(1.00)	1.33(1.00)
VEQ - facilitators			
*Self-Confidence*	1.33(1.00)	2.00(1.00)*	2.00(1.00)
*Coping with failure*	1.67(1.00)	2.00(1.00)*	1.67(1.00)
PSQI	6.0(5.0)	5.0(3.0)*	6.0(4.0)
IAT	46(22)	42(23)	42(23)

BMI, body mass index; BMR, basal metabolic rate; PAQ-A, Physical Activity Questionnaire for Adolescents; VEQ, Volition in Exercise Questionnaire; PSQI, Pittsburgh Sleep Quality Index; IAT, Young's Internet Addiction Test. *p < 0.05 vs girls. §p < 0.05 vs boys.

In girls, regarding the correlation between VEQ factors and body composition, “reasons” was positively correlated with the %FM (*r* = 0.281; *p* = 0.012), and “unrelated thought” was positively correlated with BMI (*r* = 0.215; *p* = 0.031). Moreover, correlations between VEQ inhibitors and facilitators and PAQ-A, PSQI, and IAT are reported in Fig. 1. Specifically, “postponing training” was positively correlated with PSQI (*r* = 0.198; *p* = 0.047) and negatively with PAQ-A (*r* = −0.305; *p* = 0.002), “unrelated thought” was positively correlated with PSQI (*r* = 0.220; *p* = 0.027), IAT (*r* = 0.221; *p* = 0.026), “approval for others” was positively correlated with PSQI (*r* = 0.224; *p* = 0.024) and IAT (*r* = 0.383; *p* < 0.001) (Fig. 1). Regarding the facilitator factors, “self-confidence” was negatively correlated with PSQI (*r* = −0226; *p* = 0.023) and positively with PAQ-A (*r* = 0.378; *p* < 0.001); “coping with failure” was positively correlated with PAQ-A (*r* = 0.224; *p* = 0.024) (Fig. 1).

**Fig. 1:** Correlation analyses between VEQ factors and Pittsburgh Sleep Quality Index (PSQI); Internet Addiction Test (IAT) and Physical Activity Questionnaire for Adolescents (PAQ-A) in girls. A) Correlation between Postponing Training and PSQI; B) Correlation between Postponing Training and PAQ-A; C) Correlation between Unrelated thoughts and PSQI; D) Correlation between Unrelated thoughts and IAT; E) Correlation between Approval from others and PSQI; F) Correlation between Approval from others and IAT; G) Correlation between Self-confidence and PSQI; H) Correlation between Self-confidence and IAT and I) Correlation between Coping with failure and PAQ-A.

In boys, regarding body composition variables, PAQ-A was negatively correlated with %FM (*r* = −0.306; *p* = 0.033) and “unrelated thoughts” was negatively correlated with BMI (*r* = −0.291; *p* = 0.038). PSQI was positively correlated with IAT (*r* = 0.440; *p* = 0.001). Correlations between VEQ inhibitors and facilitators and IAT are reported in Fig. 2.

**Fig. 2:** Correlation analyses between VEQ factors and Young's Internet Addiction Test (IAT) in boys. A) Correlation between Postponing training and IAT; B) Correlation between Unrelated thoughts and IAT; C) Correlation between Self-confidence and IAT; D) Correlation between Coping with failure and IAT.

Specifically, “postponing training” and “unrelated thoughts” were positively correlated with IAT (*r* = 0.510; *p* < 0.001; *r* = 0.555; *p* < 0.001, respectively), “self-confidence” and “coping with failure” correlated negatively with IAT (*r* = −0.355; *p* = 0.010; *r* = −0.465; *p* = 0.001).

The Wilcoxon Signed Rank Test revealed that body composition was not affected by the PA intervention (Table 2). No differences were observed for the PSQI, PAQ-A and IAT. The VI postponing training showed a significant decrease after the PA intervention (T_0_ = 4.5(7.0); T_5_ = 2.0(7.0); *p* = 0.003). Similarly, the VF self-confidence showed a significant decrease after the PA intervention (T0 = 6.0(4.0); T_5_ = 4.0(4.0); *p* = 0.003). The PA intervention did not affect the other volition inhibitors and facilitators (Table 2).

**Table 2:** Body composition and behavioral factors before (Pre) and after (Post) the PA intervention.

	Pre (*n* = *43*)	Post (*n* = *43*)
Age [years]	16.0(1.0)	
Height [m]	1.61(0.15)	1.62(0.15)*
Mass [kg]	60.50(18.42)	58.05(7.8)
Muscle Mass [kg]	22.65(8.62)	21.80(6.2)
Fat Mass [kg]	18.45(10.05)	18.3(5.5)
BMI [kg/m^2^]	21.60(5.34)	21.40(4.3)
Fat Mass [%]	27.75(12.82)	30.9(9.0)
BMR [kcal]	1268.50(302)	1241.50(231)
PAQ-A	1.95(0.74)	1.77(0.72)
VEQ - inhibitors		
*Reasons*	3.0(4.0)	3.0(4.0)
*Postponing training*	4.5(7.0)	2.0(7.0)*
*Unrelated thoughts*	2.0(5.0)	2.0(5.0)
*Approval from others*	3.0(4.0)	2.0(4.0)
VEQ - facilitators		
*Self Confidence*	6.0(4.0)	4.0(4.0)*
*Coping with failure*	6.0(3.0)	5.0(4.0)
PSQI	4.0(4.2)	5.0(3.8)
IAT	28(18)	27(19)

BMI, body mass index; BMR, basal metabolic rate; PAQ-A, Physical Activity Questionnaire for Adolescents; VEQ, Volition in Exercise Questionnaire; PSQI, Pittsburgh Sleep Quality Index; IAT, Young's Internet Addiction Test; *p < 0.05 vs Pre.

## 4 Discussion

This study investigated the relationship among volition in exercise, sleep quality, and internet addiction in adolescents. Moreover, here we aimed at providing novel insights regarding the effects of a school-based PA intervention on these variables. Since longitudinal studies have shown that the highest decline in PA occurs during adolescence [31], the results of this study may be helpful to increase adherence to PA programs and to counteract the later onset of the major NCDs. Our results revealed gender differences in some anthropometric parameters as well as in some volition factors, PA levels, and sleep quality. Body composition was different between girls and boys. Boys were taller and heavier than girls with a higher muscle mass and lower fat mass, thus resulting in a higher resting metabolic rate. During puberty, hormones may cause important changes in body composition in girls and boys [32]. Since our participants' age was on average 16 years old, it is reasonable that the peak of physical maturity corresponding approximately to 14 years for boys and 12 years for girls was already reached [32] Since, the rate of NCDs continues to rise, understanding the key points to reduce adolescent sedentary behavior is fundamental. Indeed, adolescence is recognized as a stage of life during which people start to adopt unhealthy lifestyles (e.g., physical inactivity, low fruit and vegetable intake, and cigarette smoking) [5]. For this reason, modifying unhealthy or unsafe behaviors during adolescence is as a primary prevention strategy for the onset of NCDs in later stages of life. Schools represent an ideal setting for the promotion of healthy habits like PA participation. Indeed, adolescents may receive positive stimuli to establish a long-lasting healthy lifestyle. However, during adolescence a decrease in PA has been reported, especially in developed countries [33]. Our results confirm a previous study showing lower PA levels in girls compared to boys as well as a greater motivation to perform PA in boys compared to girls [19]. Both psychological and motivational factors may influence the participation and the adherence to PA [17]. However, motivational process as the intention of a behavioral change may not be sufficient to explain *per se* the participation to PA. According to the Rubicon model of action phases, the cognitive processes involved in this framework include both motivation and volition [34]. As volition explains how actions are transformed into concrete actions, volitional process is essential to implement the actual behavior [18]. Our results showed for the first time that some factors of the volition in exercise questionnaire differ between boys and girls. Moreover, we showed that volitional process are correlated to internet addiction and sleep quality. Boys showed lower scores in “postponing training” and higher scores in “self-confidence” and “coping with failure” factors than girls. Interestingly, “postponing training” and “self-confidence” are the stronger predictors of hourly participation in exercise activities [18] “Postponing training” influences the transition from the pre-actional to the actional phase, where the intention is transformed into action, “self-confidence” relates to the pre-actional phase and regards the individual's trust on his/her own abilities to successfully face the challenge. All these gender differences could also account for the higher PA levels observed in boys compared to girls. Physical education teacher should consider these differences when programming a school-based physical exercise program trying to choose the optimal exercises and to give the appropriate feedback according also to gender. In girls, our results showed that reasoning about participating in PA may negatively influence the level of fat mass. Moreover, the tendency to procrastinate the PA participation, the failure to concentrate during PA, being susceptible to other people's opinions, may negatively affect the overall sleep quality. Contrarily, believing in one's own capacities may positively influence the overall sleep quality. The ability to cope with an experience of failure may positively influence the amount of PA. Finally, to be susceptible to other people's opinions may increase the level of internet addiction. Therefore, we may suppose that when PA is performed with the aim to obtain approval for others, this could lead to a bad sleep quality and high internet addiction in girls. These considerations should be taken into account, especially in the context of school-based PA or when PA is performed in group. Indeed, being susceptible to other people's opinion, may hinder the motivation towards engaging in difficult or novel exercises in front of classmates.

In boys, none of the VEQ factors correlated significantly with sleep quality. Conversely, some VEQ factors correlated with internet addiction. Indeed, the tendency to procrastinate the PA participation and the failure to concentrate during PA may increase the internet addiction levels. On the contrary, high level of self-confidence and the ability to cope with an experience of failure may reduce the time spent on internet. As expected, higher levels of internet addiction are associated with worse sleep quality. Despite the limited variance explained by the correlation coefficients, these latter pave the way for future research on a larger sample of participants. The five-month school-based PA intervention was not sufficient to improve body composition, PA levels, sleep quality and reduce internet addiction. However, for the first time we showed that a five-month PA intervention proved to be effective in reducing two subcomponents of volition in exercise, which have been related to the transition from the pre-action phase to the action phase. Specifically, the tendency to procrastinate the PA participation was lower after school based PA intervention indicating its positive effects to increase the amount of PA, especially in girls. In addition, the decrease in self-confidence after PA intervention can be accounted for by the type and method of PA performed by students. As all adolescents did the same PA program, it is conceivable that some students perceived the PA more difficult than others did, and some of them were not able to complete the requested task resulting in reduced self-confidence. According to these results, the individualization of the type of exercise according to the individual student capacities stands out as a fundamental issue. As in adolescence unhealthy lifestyle may lead to several health-related risk factors [5], PA interventions represent an important modifiable factor to work on, especially in this age group. Moreover, our results highlight the role of PA as a potential factor influencing the individual predisposition towards exercise. Therefore, school settings should be aware of the potential role of PA on volition processes during adolescence and how these latter could differ between genders in order to structure appealing PA interventions aiming to tackle sedentary behavior. We are aware of some study limitations. First, we did not re-test the entire student cohort that were enrolled in the pre-test in the study due to COVID-19 restrictions. Second, the age of our sample limits the applicability of our results to high school students. Last, we did not classify students according to their pubertal stage to better identify their biological age. Further studies are needed to analyze different school-based PA interventions according to gender and pubertal stage in a larger number of students.

In conclusion, we showed that the relationships among volition in exercise, sleep quality and internet addiction are different between girls and boys. School-based PA interventions may influence self-confidence and the tendency to procrastinate the PA participation in adolescents. Exercise specialists should consider gender differences to realize optimal PA interventions aiming at increasing self-confidence and reducing the tendency to postpone training resulting in enhanced exercise adherence to prevent the onset of NCDs.

## Ethic statement

After being informed of the aims, risks and benefits of the study, participants gave their assent and their legal guardians, in case of minors, gave their consent to participate in this study by signing the written informed consent approved by the Italian Ministry of Education (MUR; protocol number: 0005570). All the procedures detailed in the following paragraphs comply with the Declaration of Helsinki on studies on human participants.

## Disclosure statement

The authors report there are no competing interests to declare.

## Data availability statement

Dataset will be made available upon request.

## CRediT authorship contribution statement

**Francesca Greco:** Writing – review & editing, Methodology, Investigation, Data curation. **Federico Quinzi:** Writing – review & editing, Methodology, Investigation, Data curation. **Maria Cristina Papaianni:** Writing – review & editing, Supervision, Methodology, Investigation, Data curation. **Loretta Francesca Cosco:** Investigation, Data curation. **Cristina Segura-Garcia:** Writing – review & editing, Visualization, Supervision, Conceptualization. **Gian Pietro Emerenziani:** Writing – review & editing, Writing – original draft, Supervision, Methodology, Formal analysis, Data curation, Conceptualization.

## Declaration of competing interest

The authors declare that they have no known competing financial interests or personal relationships that could have appeared to influence the work reported in this paper.
